RETRACTED

# LncRNA GAS5 Interacts with MicroRNA-10b to Inhibit Cell Proliferation and Migration and Induces Apoptosis in Colorectal Cancer

**DOI:** 10.1155/2022/4996870

**Published:** 2022-01-22

**Authors:** Rui-qi Yang, Zhe-zhu Jin, San-ya Jiang, Yong-jun Jin

**Affiliations:** Zhejiang Hospital of Integrated Traditional Chinese and Western Medicine, China

## Abstract

**Objective:**

The purpose of this study was to study the effects of the GAS5/microRNA-10b (miR-10b) axis on proliferation, migration, and apoptosis of colorectal cancer (CRC).

**Methods:**

The expression levels of GAS5 and miR-10b in CRC tissues and cells were detected by quantitative real-time polymerase chain reaction (qRT-PCR). Wound healing experiment was used to detect the effects of GAS5 and miR-10b on the migration of CRC cells. The luciferase reporter gene experiment was used to verify miRNA targets. Immunohistochemical assay was used to detect the expression of proteins related to metastasis and apoptosis in tumor tissues.

**Results:**

The expression of GAS5 was downregulated in CRC tissues and cell lines. The overexpression of GAS5 can inhibit cell proliferation and progression, induce apoptosis in vitro, and inhibit the growth of CRC tumor in vivo. In contrast, the expression of miR-10b, a downstream target of GAS5, was increased in CRC tissues and cells. Suppression of the miR-10b gene can inhibit proliferation and metastasis and cause apoptosis of CRC cells. In addition, luciferase reports show that GAS5 inhibits the progression of CRC cells by binding to miR-10b. Rescue experiments showed that overexpressed miR-10b could reverse GAS5-mediated antitumor effect on CRC cells in vivo and in vitro.

**Conclusions:**

LncRNA GAS5 interacts with miR-10b to inhibit cell proliferation and migration and induces apoptosis in colorectal cancer. GAS5 and miR-10b could become potential therapeutic targets for CRC.

## 1. Introduction

Colorectal cancer (CRC) is one of the most frequently diagnosed malignant tumors in the world [1]. About 2/3 of CRC patients come from developed countries [2]. Although some genetic factors, weight, physical activity, and smoking are associated with the prognosis of patients with CRC, many patients with CRC have recurrence and metastasis. Little is known about the detailed molecular mechanism of the occurrence and development of CRC.

Long noncoding RNA (LncRNA) is noncoding RNAs with a length of more than 200 nucleotides [3]. Some LncRNAs with a size of more than 90 kb are also known as microRNAs (miRNAs). The standard “non-coding” refers to the absence of open reading frames and/or conserved codons in transcripts. The ability to encode peptides is not necessarily in conflict with the knowledge of transcripts to act as functional RNAs. In fact, there is growing evidence that bifunctional transcripts can act as both protein templates and LncRNAs [4]. More and more evidence show that LncRNAs are involved in all aspects of cell physiology and are very important for the occurrence, development, and metastasis of cancer [5]. LncRNA growth inhibition-specific gene 5 (GAS5) is located at 1q25 [6]. Several studies have shown that GAS5 is downregulated and plays a role as a tumor suppressor gene in breast cancer [7], ovarian cancer [8], hepatocellular carcinoma [9], and CRC [10]. Additionally, increasing evidence confirms that GAS5 binds to miRNAs [11]. MiRNAs are small endogenous noncoding RNA molecules (about 22 nt), which play an important role in gene expression and can promote translation inhibition or degradation [12]. Among several candidate miRNAs that regulate cell progression, a large amount of evidence has reported that the expression of microRNA-10b (miR-10b) is related to tumor growth and spread in many cancers [13, 14]. Recently, it has been reported that miR-10b promotes the cell migration and invasion in CRC tumors by targeting HOXD10 [15]. Based on the above studies, we speculate that GAS5 can regulate CRC progression by binding miR-10b, which has not been explored in previous studies. Therefore, in present study, we investigated the possible functions and mechanisms of the GAS5/miR-10b axis in CRC progression through in vivo and in vitro experiments, which may provide new ideas for CRC metastasis and treatment.

RETRACTED

## 2. Materials and Methods

### 2.1. Patients and Specimens

From September 2018 to October 2020, 50 cases of primary colon cancer tissues and adjacent normal tissues were obtained from Zhejiang Hospital of Integrated Traditional Chinese and Western Medicine. All subjects signed the informed consent form. The research was approved by the ethics committee of Zhejiang Hospital of Integrated Traditional Chinese and Western Medicine (2021-208).

### 2.2. Cell Culture

The human CRC cell lines SW480 and HCT116 were purchased from Cell Bank of the Chinese Academy of Sciences (Shanghai, China) and were cultured in RPMI-1640 (Gibco, USA) with 10% fetal bovine serum (FBS, Gibco, USA). GAS5 overexpression vector (GAS5) and empty vector, miR-10b mimics (miR-10b) and mimic NC (NC), miR-10B inhibitor (miR-10b-inh), and inhibitor NC (NC-inh) were synthesized by GenePharma (Shanghai, China). Transfection was conducted with Lipofectamine 2000 (Thermo Fisher Scientific, Inc., USA) according to the protocol.

### 2.3. Cell Proliferation and Apoptosis

Cell Counting Kit-8 (CCK-8) was utilized to detect the proliferative ability of cells. The cells were planted into 96-plates with 10000 cells per well. The apoptosis rate was observed by Annexin V-FITC/PI apoptosis detection kit. Finally, the apoptosis rate was detected by flow cytometry.

RETRACTED

### 2.4. Cell Migration Assay

Cells were added into 6-well plates and cultured to 90% concentration. Make artificial wound with 200 *μ*L pipette. In order to calculate cell mobility, appropriate time points such as 24 and 48 h after cell images were selected. Mobility (or percentage of wound healing) is the ratio of 48 h migration area (0 h–48 h scratch area) to 0 h area.

### 2.5. Quantitative Real-Time PCR (qRT-PCR)

The total RNA was extracted by the TRIzol Reagent (Invitrogen). SYBR® Premix Ex TaqTM II (Takara Bio, Shiga, Japan) was used to reverse transcribe total RNA into cDNA under the instruction guide of the manufacturer. SYBR Green Mastermix (Takara Bio, Japan) with a Step One Plus Real-Time PCR system (Applied Biosystems) was used for amplification.

### 2.6. Double Luciferase Report Experiment

Each sample has three values: RLU1-firefly luciferase reaction intensity, RLU2-internal reference sea kidney luciferase reaction intensity, and ratio-RLU1/RLU2. Generally, the ratio value can be recorded, but RLU1 and RLU2 are the actual fluorescence intensity values, which can reflect the transfection efficiency of cells, and the ratio of reporter plasmid to internal reference can also be adjusted according to the actual fluorescence intensity.

### 2.7. Immunohistochemistry Analysis

The biopsy specimens boiled 30 min in hydrogen peroxide and sealed 40 min with goat serum. The primary antibody was incubated at 4°C in serum (1RU 100) overnight. All sections were stained with 2-aminobenzidine (2-aminobenzidine) and hematoxylin (hematoxylin) for 60 min with HRP binding protein second antibody culture.

### 2.8. In Vivo Assay

16 female nude mice were subcutaneously injected into the flank of BALB/c-nu mice to develop the subcutaneous tumor bearing model. Tumor weight and tumor volume were measured every 2 days.

### 2.9. Statistical and Analytical Methods

The data are shown as mean ± standard deviation (SD). SPSS 22.0 was used for statistical analysis. *t*-test was utilized to analyze the difference between the two groups. The differences between the two groups were compared by single factor analysis of variance. *p* < 0.05 was considered to be statistically significant.

## 3. Results

### 3.1. The Expression of GAS5 in CRC Tissues and Cell Line

At first, the expression of GAS5 was detected in 50 surgical specimens by qRT-PCR. the expression level of GAS5 in cancer tissues was lower than that in normal tissues adjacent to cancer (*p* < 0.05, Figure 1(a)), and the expression level of GAS5 in CRC cell lines SW480 and HCT116 was significantly downregulated compared with that in normal colon epithelial cells NCM460 (*p* < 0.01, Figure 1(b)). Kaplan Meier (KM) curve results showed that patients with low expression of GAS5 had poor prognosis (Figure 1(c)).

RETRACTED

### 3.2. Overexpression of GAS5 Can Inhibit the Proliferation and Migration of CRC Cells

In order to elucidate the potential effect of GAS5 on CRC cells, 48 h after transfection of SW480 and HCT116 with GAS5 or vector, high expression of GAS5 (Figures 2(a) and 2(b)) was observed in the two kinds of cells. CCK-8 assay was used to detect cell proliferation. The results showed that overexpression of GAS5 inhibited the proliferation of CRC cells. In addition, flow cytometry showed that the overexpression of GAS5 could induce apoptosis (Figure 2(c)) of SW480 and HCT116 cells. The results of the scratch test showed that the cell migration ability of SW480 and HCT116 was significantly inhibited (Figures 2(d) and 2(e)) after the overexpression of GAS5. In addition, we used qRT-PCR to detect the expression of apoptosis-related gene and EMT-related gene in CRC cells after the overexpression of GAS5. It was found that proapoptotic genes such as BAK and BAX were highly expressed after the overexpression of GAS5. On the contrary, antiapoptosis-related genes Bcl-2 showed low expression. At the same time, the genes related to cell migration were also significantly downregulated after the overexpression of GAS5 (Figure 2(f)). These results suggest that the overexpression of GAS5 inhibits the proliferation and migration of CRC cells in vitro.

### 3.3. LncRNA GAS5 Targeting miR-10b in SW480 and HCT116 Cells

We used Starbase database (https://starbase.sysu.edu.cn/starbase2/index.php) to calculate the binding sites of GAS5 and miR-10b, and miR-10b was forecasted to bind with GAS5 directly in SW480 and HCT116 cells (Figure 3(a)). QRT-PCR showed that the expression of miR-10b was downregulated after the overexpression of GAS5; on the contrary, si-GAS5 transfection remarkably enhances miR-10b level in SW480 and HCT116 cells (Figure 3(b)). The subsequent double luciferase report test further confirmed the direct binding of GAS5 and miR-10b (Figure 3(c)–3(d)).

### 3.4. miR-10b Promotes the Proliferation and Migration of CRC

The expression of miR-10b was detected, the results showed that the expression level of miR-10b in tumor tissues was significantly higher than that in normal tissues, and the same result was observed in cell lines (Figures 4(a) and 4(b)). In order to accurately study the function of miR-10b, we use miR-10b inhibitor (miR-10b-inh) to specifically inhibit miR-10b.  Figure 4(c) shows the inhibition efficiency. CCK-8 assay was used to detect cell proliferation, and the results showed that miR-10b-inh inhibited the proliferation of CRC cells (Figure 4(d)). Flow cytometry showed that miR-10b-inh significantly increased the apoptosis ratio (Figures 4(e) and 4(f)) of CRC cell lines SW480 and HCT116. Wound healing test showed that miR-10b-inh inhibited the migration ability of SW480 and HCT116 cells (Figures 4(g) and 4(h)). The results suggest that miR-10b plays the role of oncogenes and maintains cell survival and metastasis.

RETRACTED

### 3.5. Overexpressed miR-10b Reverses Antitumor Effects of LncRNA GAS5 in SW480 and HCT116 Cells

Next, we further verified that the interaction between GAS5 and miR-10b regulates the proliferation and migration of tumor cells in vitro. First of all, we constructed an overexpressed cell line and verified the transfection efficiency by qRT-PCR (Figure 5(a)). MiR-10b significantly restored GAS5-reduced cell proliferation in SW480 and HCT116 cells (Figure 5(b)). And miR-10b significantly reverses GAS5-induced cell apoptosis in SW480 and HCT116 cells (Figures 5(c) and 5(d)). In addition, miR-10b reversed GAS5-induced cell migration (Figures 5(e) and 5(f)). MiR-10b inhibited GAS5-reduced metastasis and proliferation-related mRNA expression and apoptosis-related mRNA expression (Figure 5(g)).

### 3.6. Overexpressed miR-10b Reverses Antitumor Effects of LncRNA GAS5 In Vivo

HCT116 cells were cotransfected with GAS5 or vector and miR-10b or miR-NC. As shown in Figure 6(a), tumor growth in the GAS5 group was markedly slower than that in the vector group. However, the overexpression of miR-10b restored tumor growth (Figure 6(a)). Similarly, the tumor growth curve and tumor weight showed the same trend (Figures 6(b) and 6(c)). We measured the levels of ki67, BAK, Bcl-2, and E-cadherin in the tumor tissue. Compared with the vector group, the GAS5 group had downregulated ki67 and Bcl-2 expression and upregulated BAK and E-cadherin expression. On the contrary, miR-10b reversed the effect of GAS5 (Figure 6(d)). MiR-10b could obviously reverse antitumor effect of GAS5; thus, the GAS5 inhibits CRC tumorigenicity by suppressing miR-10b.

## 4. Discussion

LncRNA is a new star in the field of cancer diagnosis and treatment. Emerging evidence shows that the abnormal expression and mutation of lncRNA and SNPs are related to tumor occurrence and metastasis, affecting cancer cell proliferation, apoptosis, and EMT [16, 17]. More and more studies have reported significant changes in the expression of lncRNA in various cancer tissues, but the role of lncRNA is still controversial. Some lncRNAs play the role of promoting cancer in CRC, while others play the role of tumor suppressor. GAS5 was originally described by a potential tumor suppressor screening report with increased expression levels during growth arrest [18]. Previous studies have explored the role of GAS5 in cancer [19]. Previous reports have shown that GAS5 is underexpressed in various cancers and acts as a tumor suppressor, including CRC [20], osteosarcoma [21], and lung cancer [22]. This study revealed that GAS5 was significantly downregulated in CRC tissues and cells. Functional experiments showed that the overexpression of GAS5 could inhibit migration and proliferation of CRC cells in vitro and inhibit the occurrence of CRC tumor in viv*o*. We proved that GAS5 functioned as a tumor suppressor in CRC.

RETRACTED

It is reported that GAS5 can combine various miRNAs in some common cancers. GAS5 inhibits the proliferation of gliomas by regulating PTEN through microRNA-106b [23]. LncRNAGAS5 inhibits the invasion and proliferation of ovarian clear cell carcinoma through the miR-31-5p/ARID1A axis [24]. At the same time, other studies have shown that LncRNAGAS5 inhibits the activation of SIRT1/PGC-1a/Nrf2 signal pathway by miR-579-3p and reduces cell death in septicemia-related renal injury [25]. It is well known that the role of cell death in antitumor has become more and more obvious.

A great deal of evidence has reported that the miR-10b expression is related to tumor growth and spread in many cancers. Mir-10b plays an inhibitory role in the development of gastric cancer [26]. Zou et al. found that the downregulation of miR-10b in cervical cancer tissue and the resulting increase in HOXA1 levels may play a key role in the progression of cervical cancer [27]. Li et al. found that TUC338 may promote bladder cancer by upregulating miR-10b [28]. In this study, the expression of miR-10b in CRC tissues and cells was significantly increased and the downregulation of miR-10b inhibited the progress of CRC cells, which was consistent with previous studies. Subsequently, miR-10b is predicted to be the target of GAS5. Therefore, we further explore whether GAS5/miR-10b is related to the progress of CRC. The results show that overexpressed GAS5 plays an antitumor effect through direct interaction with miR-10b in vitro and in vivo.

## 5. Conclusion

In present study, we demonstrated that GAS5 was downregulated, and miR-10B was upregulated in CRC tissues and cell lines. The overexpression of GAS5 can inhibit cell proliferation and migration, promote apoptosis in vitro, and inhibit the growth of CRC tumor in vivo. Moreover, GAS5 exhibited antitumor effects via direct interaction with miR-10b. The regulatory network of the GAS5/miR-10b axis may provide new ideas for the metastasis and treatment of CRC.

RETRACTED

## Figures and Tables

**Figure 1:** LncRNA-GAS5 acts as a tumor suppressor gene in colorectal cancer. (a) qRT-PCR was used to analyze GAS5 level in CRC tissues. (b) qRT-PCR analysis of the LncRNA GAS5 expression in CRC cell lines and normal cell line NCM460. (c) Kaplan Meier (KM) plotter online tool was used to analyze the relationship between GAS5 expression and survival of colon cancer patients. ^∗^*p* < 0.5, ^∗∗^*p* < 0.01, ^∗∗∗^*p* < 0.001. Data represent at least three independent sets of experiment.

**Figure 2:** Biological functions of GAS5 in CRC cells. (a) Transfection efficiency of GAS5 mimic was confirmed by qRT-PCR. Cell proliferation ability (b) and apoptosis rate (c) were detected by CCK-8 assay and flow cytometry in SW480 and HCT116 cells, respectively. (d, e) Wound healing experiment. (f) qRT-PCR to detect the expression of apoptosis-related gene and EMT-related gene after overexpression of GAS5. ^∗^*p* < 0.5, ^∗∗^*p* < 0.01, ^∗∗∗^*p* < 0.001. Data represent at least three independent sets of experiment.

**Figure 3:** LncRNA GAS5 targeting miR-10b in SW480 and HCT116 cells. (a) Identification of miR-10b as a binding target of LncRNA GAS5. (b) qRT-PCR was used to detect the expression of miR-10b in SW480 and HCT116 cells after GAS5 overexpression. (c, d) Detection of miR-10b luciferase activity in SW480 and HCT116 cells. ^∗^*p* < 0.5, ^∗∗^*p* < 0.01, ^∗∗∗^*p* < 0.001. Data represent at least three independent sets of experiment.

**Figure 4:** The biological effects of miR-10b on CRC cells. The expression of miR-10b was examined in CRC tissues (a) and cell lines (b) using qRT-PCR. (c) Transfection efficiency was confirmed by RqT-PCR. Cell proliferation ability (d) and apoptosis rate (e, f) were detected by CCK-8 assay and flow cytometry. (g, h) Wound healing experiment. ^∗^*p* < 0.5, ^∗∗^*p* < 0.01, ^∗∗∗^*p* < 0.001. Data represent at least three independent sets of experiment.

**Figure 5:** Overexpressed miR-10b reverses antitumor effects of LncRNA GAS5 in SW480 and HCT116 cells. (a) Cells were constructed an overexpressed cell line and verified the transfection efficiency by qRT-PCR. Cell proliferation ability (b) and apoptosis rate (c, d) were detected by CCK-8 assay and flow cytometry. (e, f) Wound healing experiment. (g) Metastasis and proliferation-related mRNA expression and apoptosis-related mRNA expression. ^∗^*p* < 0.5, ^∗∗^*p* < 0.01, ^∗∗∗^*p* < 0.001. Data represent at least three independent sets of experiment.

**Figure 6:** Overexpressed miR-10b reverses antitumor effects of LncRNA GAS5 in vivo. (a) Represented images of tumors. (b) Tumor volumes. (c) Represented tumor weights. (d) Represented the levels of ki67, BAK, Bcl-2, and E-cadherin in the tumor tissue. ^∗^*p* < 0.5, ^∗∗^*p* < 0.01, ^∗∗∗^*p* < 0.001. Data represent at least three independent sets of experiment.

RETRACTED

## Data Availability

The data used to support the findings of this study are available from the corresponding author upon request.
